The article "The Influence of PDCA Process Management on the Incidence of Stab Wound and Psychological Anxiety of Nursing Interns" was retracted in 2023. Reasons: signs of a paper mill; compromised peer review; unreliable results or conclusions.

# The Influence of PDCA Process Management on the Incidence of Stab Wound and Psychological Anxiety of Nursing Interns

**DOI:** 10.1155/2022/8453697

**Published:** 2022-08-21

**Authors:** Meitong Chen, Dan Zhang

**Affiliations:** ^1^Department of Scientific Research and Teaching, Hubei No. 3 People's Hospital of Jianghan University, Wuhan City, Hubei Province 430033, China; ^2^Cardiovascular Medicine, Hubei No. 3 People's Hospital of Jianghan University, Wuhan City, Hubei Province 430033, China

## Abstract

**Objective:**

To research the influence of PDCA (Plan-Do-Check-Act) process management on the incidence of needle injury and psychological anxiety of nursing interns.

**Methods:**

This study belonged to the experimental study. A total of 180 nursing interns who practiced in the hospital from March 2020 to April 2022 were studied. A total of 135 interns from March 2020 to March 2021 were selected as the control group and 175 interns from April 2021 to April 2022 as the research group. PDCA process management was carried on in the research group. The control group did not make any intervention only following the routine teaching plan. The incidence of needle injury, theoretical knowledge, behavior score, self-rating anxiety scale (SAS), professional self-efficacy questionnaire score, and nursing practice satisfaction score were evaluated before and after 12 months of management.

**Results:**

After management, the incidence of needle injury in the research group was lower compared to that in the control group, and there are statistically significant differences between groups (*P* < 0.05). The scores of theoretical knowledge, attitude, and behavior in the research group were higher compared to those in the control group, and there are statistically significant differences between groups (*P* < 0.05) after management. After 12 months of management, the SAS score of the research group was lower compared to that of the control group, and there are statistically significant differences between groups (*P* < 0.05). The score of occupational self-efficacy questionnaire in the research group was higher compared to that in the control group, and there are statistically significant differences between groups (*P* < 0.05) after PDCA process management. After 12 months of management, the satisfaction score of nursing practice in the research group was higher compared to that in the control group, and there are statistically significant differences between groups (*P* < 0.05).

**Conclusion:**

Through PDCA process management, we can keep abreast of the situation of needlestick injuries among nursing students in practice and analyze in more detail the root cause of each nursing student's occupational exposure and the outcome of treatment. The nursing students not only learn more practical knowledge in clinical practice but also feel that the hospital values and cares for them, which greatly increases their satisfaction.

## 1. Introduction

Needlestick injuries are deep skin injuries caused by medical sharps such as injection needles, suture needles, and puncture needles and are one of the most common occupational risk factors faced by medical staff today [1]. The data has suggested that 80% to 90% of occupational blood-borne disease infections among health care workers are caused by needle wounds [2]. It has been confirmed that more than 20 kinds of blood-borne diseases can be transmitted by needle wounds. In the meantime, medical staff are easy to produce different degrees of psychological reactions, such as fear, anxiety, and sadness after the occurrence of needle injury. Nurses are at high risk of needle injuries as they perform daily tasks that require contact with needles such as injections and infusions [3]. However, through survey, the incidence of occupational hazards was higher among nursing students compared to nurses [4]. As future nursing staff, nursing students have to contact with all kinds of needles to complete various invasive operations every day to enhance their skills and training ability [5, 6]. However, the operation proficiency and skill level are not professional enough due to the lack of work experience. Trainee nurses are at a higher risk of unintentional injury than other medical staff, making them a higher risk group for occupational exposure in hospitals. Thus, it can be noticed that it is very important to strengthen the protection of needle stab wounds of nursing students.

PDCA theory was first put forward by Dr. Hugh Hart. Deming made a great contribution to this research [7–9]. He applied the PDCA cycle theory to many fields and put forward the idea of quality management reform, which was recognized by many management scientists and set off a new wave of quality management [10, 11]. PDCA cycle theory refers to a scientific procedure that needs to be followed in order to carry out total quality management. The content of each stage is different, and the quality management is strengthened according to the cycle order. The PDCA cycle is assigned into four stages, which is Plan⟶Do⟶Check⟶Action. P (plan) refers to the planning phase, in which the quality management plan is made according to the job requirements. D (do) refers to the implementation phase, which is carried out in accordance with the quality management plan and completes the task of quality supervision and management. C (check) refers to the inspection phase, mainly the problems that exist in the various parts of the inspection quality supervision period. A (action) refers to the processing phase, which deals with the problems summarised in the inspection phase, emphasizing the need to take into account the various influencing factors in addition to the condition of the quality control object itself, in order to inform the development of the next work plan [12]. In the 1980s, this theory was introduced into China and now it has been applied in nursing, education, medical, and other fields. PDCA process management can manage the quality of the whole training process. After many problem mining and improvement, it helps to enhance the level of training quality management and meets the quality management needs of nursing interns during their internship. Therefore, this paper considered it as the core tool of quality management research and divided the quality management of nursing interns into four stages. The influence of PDCA process management was explored on the incidence of needle injury and psychological anxiety of nursing interns.

## 2. Patients and Methods

### 2.1. General Information

The subjects were 310 nursing interns who practiced in the hospital from March 2020 to April 2022. A total of 135 interns from March 2020 to March 2021 were selected as the control group and 175 interns from April 2021 to April 2022 as the research group. There were 25 males and 150 females in the research group, aged 18 to 23 years old, with an average of 20.48 ± 0.27 years. In the control group, there were 14 males and 121 females, aged 19 to 22 years, with an average of 20.51 ± 0.31 years.

Inclusion criteria: (1) full-time nursing students; (2) cases with normal thinking, good state, and clear expression of their true feelings; and (3) willing to cooperate with this study. Exclusion criteria: (1) those who did not meet any of the inclusion criteria, (2) clinical internship nursing students who were unwilling to participate in this training due to personal factors, and (3) those with a missing value of more than 10% in the collected questionnaire.

### 2.2. Treatment Methods

#### 2.2.1. Technical Route

The technical route is indicated in Figure 1.

#### 2.2.2. Intervention Program

In the control group, the trainee nursing students received the traditional teaching mode after entering the department, including a weekly lecture. The content of lecture was based on the teaching plan designated by each department. A big lecture was organized by the Ministry of Science and Education according to the teaching progress specified by the Ministry of Science and Education. The researchers did not intervene.

In the research group, PDCA management included planning, implementation, inspection, treatment, and finding problems. All aspects of needle injury were intervened in nurses. Set up the PDCA group: the PDCA group is composed of the Ministry of Science and Education and the backbone teachers of nursing practice teaching, the head of the Ministry of Science and Education, responsible for overall planning, organization, management, quality control, and members of the group to implement the relevant content. (1) Plan: an analysis and investigation of the causes of needlestick injuries in various departments of our hospital revealed that the lack of self-protection awareness among nursing trainees, irregularities in operation, and irregularities in medical waste disposal were the main causes of needlestick injuries among nursing trainees. The study of nursing interns in school belongs to theoretical teaching, while the practice in hospital belongs to practical teaching. Nursing practice is a transition from theory to practice. Due to new contact with clinical practice, lack of proficiency in professional and technical operation, lack of solid theoretical knowledge, poor awareness of occupational protection, no systematic protection training and standard operation, and the teaching teacher is busy in work and does not strengthen supervision over the trainee students, due to these reasons, the intern students' ability to deal with emergencies and risk prevention awareness are weak, so the probability of occupational exposure is relatively high. Formulate countermeasures: strengthen the construction of nursing practice system and give full play to the role of policy guidance. Strengthen the hospital training, improve the students' awareness of prevention, and standardize the operation behavior. Strengthen the Kone management of nursing interns, bring the prevention and treatment of needle stab wounds of nursing interns into the subject education, and further establish and consolidate the protection concept of nursing interns. Strengthen the education of safety protection and safety protection equipment. (1) Guiding ideology: adhere to the guiding principle of “caring for every nursing intern,” further implement the training requirements of nursing interns, follow the system of prevention and control of nosocomial infection management, and improve the management of nursing practice in an all-round way. Improve teaching quality and teaching effect. (2) Set the goal: according to the incidence of needle injury of nursing interns in the past two years, sort out the problems, find out reasonable countermeasures, implement step by step, until the incidence of needle injury is reduced. (3) The medical staff with less than 5 years of service have relatively more occupational exposure, which is related to the lack of clinical practice experience but much practical operation, weak protection consciousness, and unskilled operation. Departments are prepared and provide necessary and accessible protective facilities, strict implementation of safety operating procedures, and implementation of standard preventive measures. Strengthen the management of clinical teaching, carry out the training of teaching teachers in the department, and improve the teaching level of teachers. (6) Improve the assessment plan and improve students' preventive knowledge and skills. (7) Carry out the drill of emergency plan for needle injury. (2) Do: standardize the system and process of handling sharp injuries for nursing trainees, instruct nursing trainees on the standardization of operations, explain the correct use of sharp boxes, make nursing trainees aware of the hazards of needlestick injuries, and develop corresponding prevention and control countermeasures. Nursing interns should pay attention to standardized operations, enhance their awareness of self-protection, strengthen training on safety knowledge and operational norms so that they understand the hazards of needlestick injuries, handle medical waste in strict accordance with the process, and regulate nurses' behavior to reduce the occurrence of needlestick injuries. Nursing trainees with needlestick injuries should be treated accordingly according to the specific circumstances of the needlestick injury and fill in the needlestick injury registration form. (1) To formulate the system of “regulations on occupational exposure management in nursing trainees' hospital,” emphasize the consciousness of responsibility, safety, and teaching and strengthen the prevention and management of needle stab wounds of nursing interns. (2) Mobilization and deployment: hold a special meeting on nursing practice teaching, actively discuss, determine the measures and plans to reduce the incidence of needle injuries, and clarify the responsible departments and the division of work. Each department held a mobilization meeting to deploy the related work. (3) Strengthen the training of nursing interns' operation-related knowledge, establish the concept of protection, and standardize the operation behavior. The prevention and treatment of needle injuries will be included in prejob training, and senior professional teachers in the department of hospital infection management will be hired to carry out prejob training for students who are admitted to hospital internship. The comprehensive training coverage rate is 100%. If you do not participate in the training, you will not be admitted to the internship. (3) Check: according to the plan and implementation steps, the head nurses of each department randomly check the implementation of their departments from time to time and analyze the existing problems. Each department examines the operation of nursing interns every month. The scientific research and teaching department cooperates with the hospital infection management department to conduct spot checks on the operation of teaching teachers and nursing interns in various departments during the teaching supervision and inspection of nursing practice every quarter. The department is well prepared and provides the necessary and accessible protective facilities and strictly implements the safety operation rules. (4) Action: the safety team of our hospital regularly carried out occupational protection knowledge training, systematically explained the protection knowledge, and the head nurse organizes nurses to study regularly, so as to make nursing interns fully aware of the harm of needle wounds and enhance their health protection knowledge. Nursing interns are required to work strictly according to the operation procedure and each nursing intern should meet the standards, standardize, train regularly and analyze cases, strengthen the protection of sharp injuries, and correctly guide the treatment methods of sharp instruments. The protective measures taken by interns to prevent infection shall follow the principle of standard prevention, and all patients' body fluids, blood, and secretions and articles contaminated by body fluids, blood, and secretions shall be regarded as infectious pathogenic substances; when medical interns come into contact with these substances, protective measures must be taken. (1) Homogenize management of the type, quantity, and location of personal protective equipment in the whole hospital. (2) Formulate safety operation procedures. (3) Establish the examination standard of safe operation. (4) The nursing teaching team leaders of each department supervise and inspect the safe operation of the teachers every week. (5) In the process of teaching, teachers standardize their own diagnosis and treatment operation behavior, play an exemplary role, and act as promoters of safety protection knowledge to ensure that trainee students can standardize diagnosis and treatment operation behavior.

### 2.3. Observation Indicators

1. The incidence of needle injury was recorded after 12 months of study management
2. The scores of theoretical knowledge, attitude, and behavior before and after 12 months of management were studied. The questionnaire was measured by the questionnaire related to stab wounds. The questionnaire was formed on the basis of referring to the questionnaires compiled by Shi Yanping, Nie Shengxiao, Liang Peirong, and other researchers, and the reliability and validity were tested. The knowledge part of the questionnaire consists of 14 items with three options of “yes,” “no,” and “unclear.” The correct answer is 1 point, and the wrong answer or unclear answer is 0. In the attitude part, there are 11 items, using the Likert 5-grade scoring method. Complete agreement, agreement, uncertainty, disagreement, and complete disagreement are assigned 5, 4, 3, 2, and 1 points, respectively. The A5-A6 reverse score, the higher the average score, the better the protective attitude. There are 16 items in the behavior part; using the Likert 5-grade scoring method, which is always, often, sometimes, rarely, and never, assign 5, 4, 3, 2, and 1 points, respectively, in which the P10-P12 reverse score, the higher the average score, the better the protective behavior
3. The scores of self-rating anxiety scale (SAS) before and after 12 months of management were assessed. SAS took standard score ≥ 50 as anxiety, 50 ≤ SAS < 60 as mild to mild anxiety, 60 ≤ SAS < 70 as moderate anxiety, and SAS ≥ 70 as severe anxiety [13]. With the increase of the score, the degree of anxiety is more serious
4. The score of career self-efficacy questionnaire before and after 12 months of management was assessed. The career self-efficacy questionnaire included 27 items in 6 dimensions: professional attitude and belief, problem-solving ability, career information collection and career planning ability, career cognition, career value, and career choice [14]. The score ranged from 27 to 135. The higher the score, the stronger the sense of professional self-efficacy
5. The satisfaction score of nursing practice after 12 months of research and management was assessed. Medical staff satisfaction scale was used to score, including work itself, work stress, interpersonal relationship, working conditions, work return, and organizational management, a total of 6 evaluation dimensions and 20 closed items [15]. The scale was scored by Likert five-level score (1~5 points). The higher the score, the better the satisfaction

### 2.4. Statistical Analysis

SPSS 23.0 statistical software was adopted to process the data. The measurement data were presented as $\bar{x}\pm s$. The group design *t*-test was adopted for the comparison, and the analysis of variance was adopted for the comparison between multiple groups. Dunnett *t*-test was adopted for comparison with the control group. The counting data were presented in the number of cases and the percentage, *χ*^2^ test was adopted for comparison between groups, and bilateral test was employed for all statistical tests.

## 3. Results

After 12 months of management, the incidence of needle injury in the research group was lower compared to that in the control group, and there are statistically significant differences between groups (*P* < 0.05), as indicated in Table 1.

### 3.1. Scores of Theoretical Knowledge, Attitude, and Behavior before and after 12 Months of Management

Before management, there exhibited no significant difference in the scores of theoretical knowledge, attitude, and behavior (*P* > 0.05). However, after 12 months of management, the scores of theoretical knowledge, attitude, and behavior in the research group were higher compared to those in the control group, and there are statistically significant differences between groups (*P* < 0.05), as indicated in Tables 2–4.

### 3.2. Scores of SAS before and after 12 Months of Management

Before management, there exhibited no significant difference in the score of SAS (*P* > 0.05). After 12 months of management, the score of SAS in the research group was lower compared to that in the control group, and there are statistically significant differences between groups (*P* < 0.05), as indicated in Table 5.

### 3.3. Scores of Career Self-Efficacy Questionnaire before and after 12 Months of Management

Before management, there exhibited no significant difference in the score of career self-efficacy questionnaire, and the difference was not statistically significant (*P* > 0.05). After 12 months of management, the score of occupational self-efficacy questionnaire in the research group was higher compared to that in the control group, and there are statistically significant differences between groups (*P* < 0.05), as indicated in Table 6.

### 3.4. Satisfaction Score of Nursing Practice after 12 Months of Research Management

After 12 months of management, the satisfaction score of nursing practice in the research group was higher compared to that in the control group, and there are statistically significant differences between groups (*P* < 0.05), as indicated in Table 7.

## 4. Discussion

The content of each stage is different, and the quality management is strengthened according to the cycle order. The PDCA cycle is assigned into four stages, which is Plan⟶Do⟶Check⟶Action. P (plan) refers to the planning phase, in which the quality management plan is made according to the job requirements. D (do) refers to the implementation phase, which is carried out in accordance with the quality management plan and completes the task of quality supervision and management. C (check) refers to the inspection phase, mainly the problems that exist in the various parts of the inspection quality supervision period. A (action) refers to the processing phase, which deals with the problems summarised in the inspection phase, emphasizing the need to take into account the various influencing factors in addition to the condition of the quality control object itself, in order to inform the development of the next work plan [5, 6, 16, 17]. With the emphasis on occupational safety and protection in nursing in China recently, the research on needlestick injuries among nursing trainees has been increasing year by year, although the incidence has tended to decrease in recent years. However, the incidence of occupational hazards is still higher compared to nurses in formal practice [18–20]. Li Chunyan took 152 nursing students who were interns in her hospital in 2006 as the research object [21]. A self-designed questionnaire was applied to conduct a retrospective survey on the current situation of needle stab wounds among nursing students. The results indicated that 101 nursing students had needle stab wounds during the internship, accounting for 66.45%. Xu Qinhong investigated the needle stab injuries of 155 nursing students in 2010 [22]. The results indicated that 88 of the 155 trainee nursing students had needle injuries with an incidence of 56.77%. A study by Chen Yan et al. on the causes of needlestick injuries and protective measures for 108 trainee nursing students showed that 90 (83.33%) had needlestick injuries [23]. A questionnaire survey was conducted by Gao Hong, among 189 nursing students in a school [24]. The results indicated that 102 nursing students had needle wounds during the practice, and the times of needle injuries were different. Dai Yali indicated that 287 of the 544 trainee nurses had needle injuries during the 8-month internship, accounting for 52.8% [25]. The study showed that 100% of nursing students had needle stab wounds during the 11-month internship period and the frequency of needle stab wounds can be as high as 4.9/person-year [26]. This paper considered it as the core tool of quality management research and divided the quality management of nursing interns into four stages. The influence of PDCA process management was explored on the incidence of needle injury and psychological anxiety of nursing interns.

In the study, Albertoni pointed out that the first semester of internship was the semester with the most stab wounds [27]. The survey results of Bao et al. showed that the incidence of needle stab wounds among nursing interns in China was about 70% [28]. The results of the study by Chen et al. showed that the incidence of needlestick injuries exhibited statistically significant differences between practice nurses with different academic qualifications. Postgraduate students had the lowest incidence rate, which is consistent with the findings of Fang et al.'s study on the relationship between needlestick injuries and education of pediatric nurses [29–31]. Shao found that the needle injuries of nursing interns were mainly caused by intravenous infusion and syringe needles, which were mainly concentrated in the index finger and middle finger of the left hand and more than half of the needle injuries occurred when the day shift was busy [32]. The incidence was higher in the first 4-5 months of the internship and then decreased gradually.

It was found that in the first week after needle injury, the main manifestations of nursing students were anxiety and fear and experienced negative emotions such as insomnia, palpitations, and nightmares [33, 34]. In view of the serious harm caused by needle injury, the relevant departments and medical staff should always pay high attention to it. At present, PDCA process management is widely adopted in clinical teaching, practice management, and nursing training in various clinical departments, showing the advantage of continuous improvement of management quality [35]. The nursing practice management can be divided into four stages, adjusting the P stage, D stage, C stage, and A stage, respectively. The new training plan is put into the practical training activities, and new problems are excavated and checked. The issues that still need to be addressed are carried forward to the next plan to form a closed-loop system that will facilitate the management goal of reducing needlestick injuries.

This study indicated that after the implementation of PDCA process management, the incidence of needle injuries of nursing interns was lower compared to that of routine teaching, and there are statistically significant differences between groups (*P* < 0.05). The scores of theoretical knowledge, attitude, behavior, professional self-efficacy questionnaire, and satisfaction of nursing practice were higher compared to those of routine teaching. The score of SAS was lower compared to routine teaching. It has been proved that the research and application value of PDCA process management on the incidence of needle stab wound and psychological anxiety of nursing interns is more significant. In addition, it has been more helpful to reduce the anxiety of nursing interns and the incidence of needle stab wounds and enhance the professional self-efficacy of nursing interns in order to make nursing interns more satisfied with their practice work [36]. This is mainly because the analysis and evaluation of the PDCA process manage the direction of quality management and refine the development of quality management. After each cycle, the quality management system has a certain degree of improvement, showing a steady upward trend. Therefore, the application of the cycle system is of great help to improve the level of quality management. In addition, PDCA process management embodies the scientific management concept of “people-oriented,” which comprehensively manages the needle wounds of interns in the process of internship. Specifically in the P stage, it analyzes the relevant factors of needle injuries of nursing students; in the meanwhile, it has a clearer grasp of the occupational exposure and treatment process of nursing students in order to formulate targeted management programs [37–39]. During stage D, nursing students are taught needlestick injury skills so that nursing students develop a positive concept of prevention. Nursing students continue to build up their knowledge of needlestick injury protection and gain a deeper understanding of needlestick injuries, thereby alleviating anxiety and improving their sense of professional efficacy. A well-established training program for nursing students on occupational exposure practices is implemented to reduce the risk of needlestick injuries to nursing students. In stage C, we can grasp the general situation of the trainees' participation in this training and lay the foundation for the next adjustment of the clinical teaching plan according to the practice of Hui nursing interns according to the evaluation results [40]. In the A stage, by comparing the effectiveness of the management program before and after improvement, the reliability of the management improvement program can be verified and a standardized process for managing nursing trainees can be developed. This study still has some shortcomings. Firstly, the quality of this study is limited due to the small sample size we included in the study. Secondly, this research is a single-center study and our findings are subject to some degree of bias. Therefore, our results may differ from those of large-scale multicenter studies from other academic institutes. This research is still clinically significant, and further in-depth investigations will be carried out in the future.

In conclusion, the influence of PDCA process management on the incidence of needle injury and psychological anxiety of nursing interns is more significant. It is more helpful to reduce the anxiety of nursing interns and the incidence of needle stab wounds, enhance the professional self-efficacy of nursing interns, and make nursing interns more satisfied with their practice work.

## Figures and Tables

**Figure 1:** Technology roadmap.

**Table 1:** The incidence of needle injuries after 12 months of management.

Grouping	Number of cases of needle injury (example)	Incidence of needle injury (%)
Control group	16	11.85
Research group	5	2.85
*χ* ^2^ value		9.763
*P* value		0.000

**Table 2:** Theoretical scores before and after 12 months of management.

Grouping	Before management (points)	After 12 months of management (points)	*t* value	*P* value
Control group	6.39 ± 0.17	9.15 ± 0.27	72.056	<0.05
Research group	6.42 ± 0.28	13.49 ± 0.65	84.731	<0.05
*tvalue*	0.828	78.503		
*Pvalue*	>0.05	<0.05		

**Table 3:** The attitude scores of the two groups before and after 12 months of management.

Grouping	Before management (points)	After 12 months of management (points)	*t* value	*P* value
Control group	32.47 ± 1.44	48.46 ± 2.27	46.492	<0.05
Research group	32.53 ± 1.37	50.22 ± 3.17	56.579	<0.05
*tvalue*	0.297	14.245		
*Pvalue*	>0.05	<0.05		

**Table 4:** The behavior scores of the two groups before and after 12 months of management.

Grouping	Before management (points)	After 12 months of management (points)	*t* value	*P* value
Control group	45.43 ± 1.29	60.46 ± 2.44	41.613	<0.05
Research group	45.39 ± 1.32	74.48 ± 3.06	52.165	<0.05
*tvalue*	0.302	23.948		
*Pvalue*	>0.05	<0.05		

**Table 5:** Score of SAS before and after 12 months of management.

Grouping	Before management (points)	After 12 months of management (points)	*t* value	*P* value
Control group	58.25 ± 6.19	52.68 ± 4.24	6.933	<0.05
Research group	58.28 ± 6.17	43.75 ± 2.04	19.287	<0.05
*tvalue*	0.135	21.013		
*Pvalue*	>0.05	<0.05		

**Table 6:** Scores of occupational self-efficacy questionnaire before and after 12 months of management.

Grouping	Before management (points)	After 12 months of management (points)	*t* value	*P* value
Control group	71.59 ± 4.06	88.18 ± 6.11	22.508	<0.05
Research group	71.63 ± 4.13	119.53 ± 8.24	46.775	<0.05
*tvalue*	0.126	27.186		
*Pvalue*	>0.05	<0.05		

**Table 7:** Satisfaction score of nursing practice after 12 months of research management.

Grouping	After 12 months of management
Control group	90.59 ± 2.32
Research group	95.36 ± 4.14
*tvalue*	10.624
*Pvalue*	<0.05

## Data Availability

The datasets used and analyzed during the current study are available from the corresponding author upon reasonable request.
